RETRACTED

# Quality Control in the Clinical Medical Laboratory Based on Mobile Medical Edge Computing

**DOI:** 10.1155/2022/1688882

**Published:** 2022-09-27

**Authors:** Guorong Wang, Yukun Xue, Jie Lv

**Affiliations:** ^1^Clinical Laboratory, Yinan County People's Hospital, Linyi 276000, Shandong, China; ^2^Medical Laboratory Specialty, Binzhou Medical College, Binzhou 256600, Shandong, China; ^3^Clinical Laboratory, Pingyi County Traditional Chinese Medicine Hospital, Linyi 273300, Shandong, China; ^4^Clinical Laboratory, People's Hospital of Rizhao, Rizhao 276800, Shandong, China

## Abstract

Today, the IT departments of many healthcare organizations are suffering from data storage and network speed. Doctors diagnose patients to help them out, and this treatment process needs to be well managed. Clinical trial data are the main basis for judging the patient's condition in the medical process. With the rapid development of clinical laboratory technology in China, important achievements have been made in medicine. Clinical hospitals use a large number of different types of testing reagents and equipment, and the accuracy of testing data has become a key issue for testing results. The accuracy of testing data comes from the zero error of clinical testing, derived from the rigor and operational rigor of the testers in clinical testing. This article is dedicated to the quality control analysis and research based on mobile medical edge computing in clinical trials. This article introduces the relevant theories of mobile medical edge computing technology and quality control methods, with reference to the study on the general medical students' clinical competency in problem-solving, communication skills, procedure, history, and physical examination and critical and non-critical indicators in objective structured clinical examination (OSCE). In addition, a routine testing group and a quality control group for strengthening important aspects of medical testing were designed to conduct comparative experiments. Experiments have proved that the quality control group for strengthening the important links of medical testing has a higher index than the routine testing group in all aspects. Among them, the detection accuracy rate can reach up to 99.48%, which is of great significance for the improvement of the detection link of the patient's condition and the follow-up diagnosis and treatment link.

## 1. Introduction

With the rapid development of mobile communication systems and Internet technology, the demand for high-speed mobile network services in clinical testing and the rapid development of commercial traffic in the network have greatly affected and restricted the existing mobile communication architecture. To offset the impact of big data traffic on the mobile communication network, popular content can be cached at the edge of the network when the traffic is not at a peak. Mobile medical edge computing takes network connectivity and IT computing capabilities as the entry point to provide rich, low-latency edge applications and build cloud, network, edge, end industry integrated service capabilities to empower the medical industry, effectively reducing transmission latency and improving computing efficiency. Distributed caching technology can effectively reduce the transmission of unnecessary content in the network during the search process by intelligently storing service content close to the terminal, reduce network traffic, and improve network service experience.

RETRACTED

Clinical medical tests are common clinical medical operations that can provide accurate reference data for disease diagnosis and treatment. The quality control of clinical testing is first of all to ensure the accuracy of the test data. Although clinical medical trials play a very important role in clinical research, judging from the current status of clinical research in China, in terms of both hospital facilities and industrial production, they are in a backward position and are in urgent need of improvement. The establishment and operation of a complete hospital quality assurance system require complete quality control. Clinical testing is based on human factors. The whole process includes more complicated factors such as sociology, psychology, practice, and probability. The results directly affect people's life and health. Therefore, quality control throughout clinical trials is an important way and means to ensure the accuracy of the final trial data and to protect the safety and rights of subjects and has important practical significance.

To understand the current status of chemotherapy cancer treatment quality check in Beijing hospitals, the issues of major existence are identified, and the next steps are developed. Qiu et al. reviewed one clinical chart of oncology chemotherapy per month for quality control check and randomly selected 10 clinical charts from each hospital. A total of 756 patient histories from 76 hospitals were reviewed. The results of the analysis showed that the overall improvement and quality control of oncology chemotherapy met clinical standards. The Intravenous Drug Supply Service (PIVAS) was available in only 36.8% of the institutions. Oncology was higher than other departments in chemotherapy and drug quality control (*P* < 0.01). Hospitals with clinical specialists had chemotherapy and drug quality control scores of 50.6 and 14.5, respectively, higher than those without specialists at 47.2 and 12.7 (*P* < 0.05).Therefore, secondary hospitals should pay attention to the effective control of tumor chemotherapy and strengthen the training of chemotherapy personnel, but the implementation is more cumbersome [1]. An ultra-high performance liquid chromatography-evaporative light scattering detection method for fingerprint analysis of Gusprin tablets was established by Wang et al. For the detection, the nitrogen pressure was 0.28 MPa, the drift tube temperature was 60°C, and the gain was 400. 39 batches of samples from 6 manufacturers were determined by the above method, and the peaks existing in more than 75% of the cases were defined as frequent peaks, and a total of 30 common peaks were determined. The similarities of the tested samples varied from 0.47 to 0.98, showing that the quality of these samples varied significantly from one sample manufacturer to others. The results showed that some manufacturers may have problems with the breeding of Baishao, Panax notoginseng, and Wei Ling Xian. This research provides a basis for the overall quality control of Guspur tablets and the improvement of quality standards, but it has not yet been specifically applied [2]. The use of the Objective Structured Clinical Examination (OSCE) as an assessment tool has been introduced in many medical schools. The Objective Structured Clinical Examination (OSCE) is not a specific assessment method; in fact, the OSCE only provides an objective, structured, and organized assessment framework in which each medical school, hospital, medical institution, or examination body can add appropriate assessment content and assessment methods according to its own syllabus and examination syllabus. Müller details the present state of implementation of the OSCE evaluation in Germany. The status of implementation of the OSCE in all 36 German medical schools was investigated through a semi-structured. The implementation of this assessment format includes most clinical performance records, but more than half (51.4%) include surgery, internal medicine, emergency, anesthesiology, and orthopedics. The results of the report confirm the wide application of OSCE assessments in German medical schools. To ensure that physicians in the future have a wide range of clinical capabilities, the application scope of OSCE should be expanded. For this reason, further information is still needed to convince the staff of the medical school [3]. Although in the process of medical education, in order to solve the difficult transition from classroom learning to clinical training, there are various curriculum advancements, obstacles still exist. In Butts et al. DO's research, the Philadelphia College of Osteopathic Medicine (PCOM) designed a four-week course to make this transition easier to determine whether PCOM students have improved their comfort and readiness after participating in the 4-week clinical transition course before serving as third-year clinical clerk and to determine whether the teacher's awareness of student readiness and comfort has improved compared with the previous third-grade students. The course includes 16 group exercises, all of which are done before students start the third-year staff rotation. The exercises in the course went beyond the skills they learned in class. The students conduct surveys before and after class to evaluate the comfort of their 58 different aspects of clinical practice, but the practicality is not great [4]. A mobile medical unit (MMU) is a customized vehicle equipped with medical equipment to provide primary care in a rural environment. Because MMUs can be easily repositioned, they can be demand-oriented and flexibly provide local health services. Busing studied the strategic planning of MMU services, by determining where the MMU operating sites should be located and how often these sites should provide services. For this reason, the strategic planning problem of MMU (SPMMU), a set coverage problem with limited capabilities, is studied, and an integer linear programming is proposed for SPMMU, but the experimental scheme is a bit complicated [5]. As mobile edge computing (MEC) is widely used, MEC is becoming a way to narrow the gap between the healthcare workers and the doctors. Related to this, MEC is also moving towards the direction of monitoring personal health in an automated and intelligent way. Wan et al. designed a HAR architecture based on the smartphone inertial accelerometer. As players engage in similar typical everyday tasks, the sensory data mobile phone gathers a sequence of features, extracts valid traits out of the initial data, and acquires data on the user's bodily movements through several triaxial sensors. The design of the system is performed by preprocessing the actual data through noise removal, localization and splitting, and extraction of valuable characteristic vectors. He discussed how to train deep learning methods and showed how the proposed method is better than other methods on two large public data sets: UCI and PAMAP2, but the experimental data are too general [6]. Recently, with the popularization of information and communication technology (ICT) in the medical field, leading to the medical Internet of things, new electronic medical services are being provided, especially to the elderly who need daily assistance. Cisotto et al. researched and identified the top iconic healthcare cases that would potentially benefit and integrate the communication needs in these concrete cases from 5 G-enabled networks. In a representative case study of connected ambulances, the effects of taking on three key 5 G enabling technologies will be discussed, namely healthcare network slicing, cellular edge computing, and managing heterogeneous networks, but at no small initial investment cost [7]. These studies provide a detailed analysis of the quality control of clinical medical testing sessions. However, there are relatively few studies incorporating mobile edge technologies that are not thorough enough, and there is a need to fully apply these technologies in this field.

RETRACTED

This article aimed to conduct a comprehensive analysis, summary, and research on the current status of clinical trials in *S* Central Hospitals. Through the comparison and demonstration of related factors, we can further understand the main problems in the quality of clinical research and explore improvement measures. As a result, the establishment and operation of the quality assurance system can be better promoted, and effective methods to improve the professional skills of clinical researchers can be obtained more effectively. At the same time, higher requirements and standards are put forward for related inspection links, which lays a solid foundation for promoting the improvement of management level and perfecting the quality supervision system, to further do the work of clinical trials.

## 2. Quality Control Analysis Method Based on Mobile Medical Edge Computing

### 2.1. Mobile Medical Edge Computing Technology

Mobile edge computing (MEC) uses wireless access networks to make it more convenient for users to surf the Internet. MEC is a new technology based on the 5 G evolution architecture proposed by the global standard organization ETSI. Its existence provides technical support for the development of intelligent cache distribution. MEC provides users with distributed computing space and storage services in wireless networks. MEC aims to reduce network compression by shifting computing load from core cloud data to the mobile edge [8]. MEC can enable these MEC devices sent to the edge of the network to provide computing and storage services for mobile terminals in the user's area. The devices sent to the edge of the mobile network are called MEC servers. By storing multimedia content in the local MEC server in advance, users can download the required content directly from the local cache, thereby reducing unnecessary transmission, saving bandwidth resources, obtaining faster performance results, and performing higher medical examinations [9, 10].

RETRACTED

A mobile user in a wireless network close to the wireless network uses mobile edge computing to deliver IT services and cloud computing services, as shown in Figure 1. MEC can provide high-latency bandwidth-efficient service zones at the edge of the WLAN for both application development and content providers. They can get real-time access to wireless network information (e.g., user status and cell load) straight from the MEC system. It is seen that mobile edge computing could improve and enhance the user experience by providing computing resources to increase the speed of content distribution and the responsiveness of both services and the applications [11].

Along with the fast evolution of mobile communication technology, its applications in various industries are becoming wider and wider. Among them, mobile medicine developed in recent years is to provide users with medical services and information through mobile communication technology and equipment. Its most prominent feature is that it can provide pervasive health care anytime and anywhere. For example, the direct use of mobile phones can be used to support medical services. It provides a key platform for the public, which can be used as an effective service tool to determine the real-time delivery, access, and storage of health information [12]. However, the adoption of mobile device-based healthcare services faces some challenges, such as the storage capacity, security, and access control limitations of the user's use of the device.  Figure 2 shows the flow pattern of the connection configuration between the mobile client and the server.

The basic steps for the communication between the mobile phone client and the Web server are as follows: (1) the client application receives the data that need to be sent to the server, such as user account information, creates a URL, and uses the data received as a parameter in the login address [13]; (2) it uses the above URL item to set an HttpURLConnection link object and set connection parameters, including link expiration settings and query status (publishing or receiving) settings; (3) the connection object uses connect() to initiate a URL link request. If the query string is blocked, it will be processed and eliminated. Otherwise, the server will respond to the query and process it, while returning the data content [14]; and (4) the client stores the data content from the server in the BufferedReader object and executes the data function through the object.

Mobile network operators (MNOs) send multiple MEC service applications to the network edge and may send multimedia traffic (video/Web) traffic to local MEC servers in advance. Users can directly reduce network traffic by downloading the content from the neighborhood [4].

RETRACTED

The collaborative cache storage under MEC service infrastructure is illustrated in Figure 3. MNOs enable MEC servers to run on each LTE base station (Evolved Node B, eNB), thus adding computing, storage, and service capabilities to LTE wireless networks and enabling open-source applications. Open wireless networks through wireless APIs and information exchange between servers upgrade the conventional LTE cell sites to smart cell sites [15].

As shown in Figure 3, the remote central cache server and the MEC server communicate through a reverse link to distribute service content to each local cache. Area caches *c*_1_, *c*_2_, and *c*_3_ form a collaborative cache space. BSs have an integrated cache site connected via optical fiber so that MECs can communicate with each other, collaborate with each other, and be aware of shared content [16].

As shown in Figure 4, the MEC server can provide cloud services for mobile users in the Wi-Fi access point area [17]. At present, the demand for computing and storage sources of applications installed on terminal devices is increasing.

The current rapid increase in mobile users has led to the rapid growth of mobile equipment, which requires the introduction of large-scale MEC systems to transfer computing cache data from the cloud to the edge of the network, thereby alleviating the problem of global computing sources and reducing network bandwidth [18]. It can transfer the user's work data from the mobile terminal to the cloud to solve the data storage problem of the terminal device.

Because when designing the working algorithm of the MEC system, the delay time to complete the task and the amount of computing resources required are the main factors that need to be considered. Therefore, if the availability of multiple tasks before scheduling tasks is prioritized, the tasks are divided into multiple clusters with special priorities and the tasks are executed in the clusters with the first priority. Execution is completed within the tolerance period, and a less complicated task can be done first to reduce the waiting time for subsequent tasks [19, 20]. Therefore, this goal is mainly to pay attention to the cluster problem before formulating the work plan, that is, to fully plan the workload of completing tasks and the sustainability of tasks in different tasks and queues. The local SDN server in the MEC system architecture analyzes the cache. Packing tasks before building a cluster can combine tasks and is most sensitive to the computational load needed to finish them. After that, the SDN manager essentially also performs tasks in the cluster. It can be calculated first, thereby effectively reducing the queuing delay of subsequent activities.

RETRACTED

A clustering algorithm is a statistical analysis method to study the classification problem (of samples or metrics) and is also an important algorithm for data mining. The classification of clusters algorithm has been the most widely studied and applied in unsupervised learning. The most common method used in clustering algorithms is to determine the relative differences among points using the Euclidean distance of two points and the Mahalanobis distance, and the explicit distance is a generalization of the Marxist distance. The Euclidean space in n dimensions can be denoted as follows:

(1) $$\begin{array}{c} s_{1}=\sqrt{\sum_{i=1}^{n}{\left(x_{i}-y_{i}\right)}^{2}.} \end{array}$$

The Mahalanobis distance can be expressed as follows:

(2) $$\begin{array}{c} s_{1}=\sum_{i=1}^{n}\left|x_{i}-y_{i}\right|. \end{array}$$

The Marxist distance it is not affected by the dimension, and the Marxist distance between two points is independent of the measurement units of the original data and also excludes the interference of the correlation between variables.

Ming's distance can be expressed as follows:

(3) $$\begin{array}{c} s_{1}={\left(\sum_{i=1}^{n}|x_{i}-y_{i}{|}^{p}\right)}^{1/p}. \end{array}$$

Suppose at present one has *N* tasks, the numbers are {*P*_1_, *P*_2_, ..., *P*_*N*_}, while the overall computation volume completed per task corresponds to {*Q*_1_, *Q*_2_, ..., *Q*_*N*_}. Let us pretend that the task latency sensitivity of all jobs might be classified into *X* classes, denoted as {1, 2, ..., *X*}, and the delay sensitivity of *Y* tasks can be expressed as {*R*_1_, *R*_2_, ..., *R*_Y_}, where *R*_*i*_ ∈ {1, 2, ..., *X*} and *i* = {*P*_1_, *P*_2_, ..., *P*_*Y*_}. Let us categorize the groupings as {*V*_1_, *V*_2_, ..., *V*_k_}.

Assume the tasks in the SDN director at a given point in time are {*P*_1_^*∗*^, *P*_2_^*∗*^, ..., *P*_*Y*_^*∗*^}, while the relative sensitivity of the latency is {*R*_1_′, *R*_2_′, ..., *R*_Y_′}, respectively. After the delay response sensitivity is normalized, the result is {*R*_1_^*∗*^, *R*_2_^*∗*^, ..., *R*_*Y*_^*∗*^}, where

(4) $$\begin{array}{c} R_{i}^{*}=\frac{R_{i}^{'}}{{\sum^{}}_{j=1}^{n}R_{j}^{'}}. \end{array}$$

The overall computing volume necessary to finish the job is {*Q*_1_′, *Q*_2_′, ..., *Q*_Y_′}, and the result after the normalization operation is {*Q*_1_^*∗*^, *Q*_2_^*∗*^, ..., *Q*_Y_^*∗*^}, where

(5) $$\begin{array}{c} Q_{i}^{*}=\frac{Q_{i}^{'}}{{\sum^{}}_{j=1}^{n}Q_{j}^{'}}. \end{array}$$

Let us now define that the Euclidean distance among the missions *P*_*i*_^*∗*^, *P*_*j*_^*∗*^within a single agglomerate may thus be given as follows:

(6) $$\begin{array}{c} s_{2}=\sqrt{{\left(R_{i}^{*}-R_{j}^{*}\right)}^{2}+{\left(Q_{i}^{*}-Q_{j}^{*}\right)}^{2}.} \end{array}$$

Then, its average value can be expressed as follows:

(7) $$\begin{array}{c} \bar{s}=\frac{{\sum^{}}_{i=1}^{n}{\sum^{}}_{j=1,j\neq i}^{n}s_{2}}{V_{n}^{2}}. \end{array}$$

The normative error associated with those tables in cohort with *D* is defined. When there is task {*P*_1_^*∗*^, *P*_2_^*∗*^, ..., *P*_*Y*′_^*∗*^} in cluster *V*_*i*_,

(8) $$\begin{array}{c} D_{i}=\sqrt{\frac{{\sum^{}}_{i=1}^{n^{'}}{\sum^{}}_{j=1,j\neq i}^{n^{'}}\left(s_{2}-\bar{s}\right)}{V_{n^{'}}^{2}}}. \end{array}$$

By the time it is possible for all missions to be partitioned into *k* clusters, we expect results of

(9) $$\begin{array}{c} \text{min}\left\{\text{max}D_{i}\right\},i=1,2,3,...,k. \end{array}$$

Resource utilization standard deviation (RUSD) represents the discrete degree of multidimensional resource utilization on the mobile edge computing server. The smaller its value, the more balanced the utilization of various resources. The calculation formula for the standard deviation of resource utilization of the *i*th MEC server is shown in the following formula:

(10) $$\begin{array}{c} s_{RUSD}=\sqrt{\frac{1}{N}\overset{N}{\underset{n=1}{\sum }}{\left(p_{i}^{k}-p_{i}^{\prime }\right)}^{2}.} \end{array}$$

Among them, *p*_*i*_^*k*^ represents the utilization rate of the *k*th dimension resource on MEC server *i*, and *p*_*i*_′=1/*N*∑_*n*=1_^*N*^*p*_*i*_^*k*^ represents the average resource utilization rate of MEC server *i*. The resource balance rate *RB* (resource balance) needs to be used to limit the excessive utilization of resources in a certain dimension. The calculation formula for the resource balance degree of the *i*th MEC server is shown in the following formula:

(11) $$\begin{array}{c} t_{RB}=\frac{p_{i}^{'}}{{\text{max}}_{n\in \left\{1,2,...,N\right\}}p_{i}^{k}}. \end{array}$$

In formula (11), the value of *t*_*RB*_ is less than or equal to 1, *p*_*i*_′ represents the average value of the multidimensional resource utilization of the MEC server, and max_*n*∈{1, 2, ..., *N*}_*p*_*i*_^*k*^ represents the maximum value of the multidimensional resource utilization. When *t*_*RB*_ is close to 1, it means that the effect of restricting a certain kind of resource utilization is better.

RETRACTED

Resource Utilization Balance Deviation (RUBD): considering the resource utilization standard deviation RUSD and the resource balance (RB) rate, the resource utilization balance of the *i*th MEC server is expressed as follows:

(12) $$\begin{array}{c} U_{RUBD}=\frac{s_{RB}}{t_{RUSD}}. \end{array}$$

The formula for calculating the resource utilization of the *i*th MEC is shown as follows:

(13) $$\begin{array}{c} A_{RUBD}=\frac{A_{i}^{RUBD}-U_{RUBD}}{U_{RUBD}}. \end{array}$$

When the value of *A*_*RUBD*_ is greater than zero, it means that the resource utilization of the *i*th MEC server will increase; otherwise, it will decrease.

### 2.2. Quality Control Methods

#### 2.2.1. Basic Theory of Quality Control

Quality control in English is internal quality control (IQC). Quality control refers to factors directly related to analysis and measurement experiments, such as material use and measurement methods. Quality assurance focuses on monitoring the indications and results of treatment. It is one of the tasks of the testing room staff to regularly assess the reliability of the indoor testing and determine whether the report has been issued. In the normal operation of the laboratory, the consistency of the test between batches and intra-batch samples in routine work is used to determine whether the test results are reliable and whether a report can be issued. The indoor quality control part is an important part of the inspection link in the testing room, and the relationship between them and the quality assessment is shown in Figure 5.

#### 2.2.2. Quality Control Chart

Random Error: it is an inaccurate and random error caused by many uncontrollable factors.

System Error: it is an error generated during the test, and its value is either a constant or it follows a conversion rule. The cause is always a known or possible event. Therefore, as much system error as possible is predicted, and it is eliminated or controlled through careful research and design and strict technical measures.

Low Probability Event: a random probability event is between 0 and 1, which is 0 ≤ *P* ≤ 1. Most decision-making comes from probabilistic decision-making, which has a certain degree of reliability and statistical significance. Traditionally, *P* ≤ 0.05 is called a low-probability event, which means that the probability of an event being tested or observed is very small, and may be considered impossible to happen or exist.

Sample Mean: the average of all values in a set of values is as follows:

(14) $$\begin{array}{c} \bar{x}=\frac{\sum_{i=1}^{n}x_{i}}{n}. \end{array}$$

Sample Standard Deviation: it refers to the distribution of a set of data and is calculated as follows:

(15) $$\begin{array}{c} s=\sqrt{\frac{\sum^{}{\left(x-\bar{x}\right)}^{2}}{n-1}}=\sqrt{\frac{n\sum^{}x_{i}^{2}-{\left(\sum^{}x_{i}\right)}^{2}}{n\left(n-1\right)}}. \end{array}$$

Coefficient of Variation: it is expressed as a percentage of the standard deviation and its mean.

(16) $$\begin{array}{c} W=\frac{s}{\bar{x}}\times 100\text{\%}. \end{array}$$

Normal Distribution: suppose the probability density of continuous random variable *δ* is as follows:

(17) $$\begin{array}{c} f\left(x\right)=\frac{1}{\sqrt{2\pi }\sigma }e^{{\left(x-\mu \right)}^{2}/2\sigma^{2}}\left(-\infty <x<+\infty \right), \end{array}$$

where *μ*, *σ*(*σ* > 0) is a constant, and it is said that *δ* obeys the normal distribution or Gaussian distribution with a parameter of *μ*, *σ* and id recorded as *δ* ~ *N*(*μ*, *σ*^2^).

RETRACTED

The area under the normal curve has a certain distribution law, as shown in Figure 6.

Suppose the test is based on a small probability. The so-called principle of small probability refers to low-probability events that are impossible to occur in sampling inspection.

Let the test statistics be

(18) $$\begin{array}{c} Q=Q\left(x\right). \end{array}$$

*Q* is a function of the sample value and the estimated parameter. When the null hypothesis *L*_*o*_ holds, the probability density function *g*(*Q*) of the test statistic *Q* is known.

The probability of *Q* falling in a certain area *ω* is as follows:

(19) $$\begin{array}{c} P\left(Q\in \omega \right)={\int^{}}_{Q\in \omega }g\left(Q\right)dQ=M. \end{array}$$

The value of *M* is usually very small, such as *M* = 0.01 and 0.03. The mistake of rejecting the initial postulate while the original hypothesis is true is called the first type of error in hypothesis testing, and (1 − *M*) is also called the error of throwing out truth. For the type *I* error in hypothesis testing, the likelihood of making a correct decision when the null hypothesis is true is taken as the probability. The significance level is a warranty to limit the type I error and is also called the loss of the test.

In hypothesis testing, another type of error may also be made; that is, the original hypothesis is inaccurate and the original hypothesis *L*_*o*_ is incorrectly accepted. This type of error is called the second type of error in hypothesis testing. The probability of making the second type of error is denoted as *N*. Even if the null hypothesis *L*_*o*_ is incorrect, the statistic *Q* value obtained by a sampling inspection has a certain probability to fall in the (*W* − *w*) area, and then,

(20) $$\begin{array}{c} P\left[Q\in \left(W-w\right)\right]=1-P\left(Q\in \omega \right)=N. \end{array}$$

In the formula, *W* is the area of all possible values of the statistic *Q*. The schematic diagram of the two types of errors in hypothesis testing is shown in Figure 7.

As shown in Figure 7(a), the decrease in *M* reduces the probability of making the first type of error, while at the same time *N* increases, which increases the probability of making the second type of error, and vice versa. The comparison between the inspection decision and the two types of errors is shown in Table 1 (the first type of error is expressed as 1, and the second type of error is expressed as 2).

RETRACTED

Figure 7(b) shows the relationship between the loss caused by the application error of the quality control chart and the size of the control end. The minimum value is 3*σ* as the control limit. At this time, the loss caused by the application error of the quality control chart is the smallest, so the state at 3*σ* is called the most economical principle.

CUSUM quality control is a frequently used quality control method. The purpose of using clinical laboratory quality control in hospitals is to monitor the measurement process, because appropriate quality control methods can be implemented to warn analysts when abnormal conditions occur.

CUSUM quality control rules are also determined on the basis of average $\left(\bar{x}\right)$ and standard (*s*). Common quality control rules and their meanings are shown in Table 2.

## 3. Design Experiments Based on Mobile Medical Edge Computing in Clinical Medical Testing

This study adopts the stratified cluster sampling method. A total of 200 questionnaires were issued to the S Central Hospital at the two levels of internal medicine and surgery, of which 50 were issued for internal medicine and 50 were recovered, with a recovery rate of 100%. The surgical department issued 50 copies and recovered 50 copies. The recovery rate was 100%. In this study, a total of 100 valid questionnaires were recovered. The contents of the questionnaire mainly include the informed consent of the surveyed person, subject compliance, whether the investigator has enrolled subjects in strict accordance with the trial protocol, whether the clinical trial data are recorded in a standard manner, whether the laboratory abnormal value review is timely and effective, and whether the subjects participate in follow-up on time, which are the main content, as shown in Table 3.

It can be seen from Table 3 that from the perspective of the rigor of clinical medicine, the branches of each evaluation section are not very ideal. At present, the researcher's compliance item has the highest score, reaching 75 points. However, the lowest score of the subjects' compliance reached only 12 points. Every quality influencing factor of the clinical medical test has exposed many problems, which shows that the current status of the clinical medical test of the hospital is not optimistic.

This article selects the cases of S Central Hospital in the second half of 2020, takes patients who have undergone clinical medical tests as the research objects, and randomly arranges them into two groups: the routine testing group and the quality control group for strengthening the important links of medical testing. The experimental subjects were between 30 and 60 years old, and the average age of the two groups was 35 years. The number of patients in each department is shown in Table 4. Among them, the routine testing group only accepts routine medical examinations, and the specific requirements of the quality control group for the strengthened clinical medical testing are reflected as follows:

1. The director of the quality control office and the person in charge of this study will conduct joint training for clinicians who perform RCT, with special emphasis on the purpose, importance, and precautions of this study. Choosing a dedicated and cooperative doctor as the investigator, the investigator is asked to explain the importance and anonymity of the research to the test subjects, and the investigation after the patient agrees is conducted.
2. A second check on the patient information before the test is performed, and the inspection of the laboratory equipment and the state of the test object during the check are paid attention.
3. The data are entered twice to ensure that the entry is correct.

RETRACTED

## 4. Quality Control Analysis

Figure 8 shows the distribution of gender and age of patients undergoing clinical medical examinations in S Central Hospital in the second half of 2020. Through the comparative experiment of clinical medical detection of known 6-month visiting patient cases, the SPSS 21.0 statistical software is used to analyze the data, and the detection rate and detection accuracy rate of the patient's condition are shown in Figure 9. The patient's satisfaction with the inspection work and the medical staff's satisfaction with the inspection work are shown in Figure 10.

It can be seen from Figure 8 that, except for October, there are more male patients than female patients, and the age distribution of patients is regular. Generally speaking, the number of people in the 31–40 age group is the most concentrated, and the percentage of people in the 20–30 age group is the lowest.

It can be seen from Figure 9 that in the 6-month routine detection group, the detection rate of patients' conditions is relatively high, and there are some errors in the collection of samples, experimental equipment, etc., which may cause the detection rate to fail to reach 100%. However, compared with the group to strengthen the quality control of important aspects of medical testing, the monthly detection rate is still not accurate enough. The group of strengthening the quality control of important aspects of medical testing has reached 100% for three consecutive months. Compared with the detection rate, the detection accuracy rate of the patient's condition is more important. In this regard, the quality control group for strengthening the important links of medical testing is also higher than the routine detection group, up to 99.48%. This is of great significance for the improvement of the detection link of the patient's condition and the follow-up diagnosis and treatment link.

RETRACTED

It can be seen from Figure 10 that whether from the perspective of patients or medical staff, the satisfaction of the quality control group that strengthens the important links of medical testing is higher than that of the routine testing group. The satisfaction of the quality control group for strengthening the important links of medical testing is above 90%, while the satisfaction of the routine testing group is between 80% and 90%.

## 5. Conclusion

Nowadays, the mobile Internet and smart terminals are developing faster and faster, and they have penetrated all corners of society, and new mobile medical and health information service models have emerged. After the mobile edge computing solution is implemented, it can provide high-quality data connection services for customers in the medical industry by relying on its IT capability and self-service capability and provide an underlying application platform for customers based on MEC to support various hospital businesses and help hospitals achieve intelligence and informatization. Establishing a relatively complete quality assurance and quality control system for clinical medical testing is the basis for ensuring its process standardization, data reliability, and result authenticity. At the same time, it is also a crucial basis for evaluating the quality of clinical medical tests and whether clinical interventions are safe and effective. Through the comparison experiment between the routine testing group and the quality control group of the important part of the strong medical test, it can be found that the accuracy and reliability of the test results of the quality control group for strengthening the important links of medical tests have been greatly improved, which is of great help to the subsequent effective diagnosis and treatment of patients. At the same time, it can also be found in the experiment that the detection accuracy and job satisfaction are still not perfect, which is not friendly to the target patient, so it needs to be improved in the following aspects: (1) before deciding on the experimental plan, medical professionals should also interact and communicate well with patients. A good attitude will help the inspection process proceed smoothly. (2) The hospital can implement digital control and management for inspection and diagnosis and regularly maintain and inspect the facilities to ensure that all facilities and instruments are in good condition.

RETRACTED

## Figures and Tables

**Figure 1:** MEC system architecture diagram.

**Figure 2:** Connection flowchart between client and server.

**Figure 3:** Cooperative content caching system model based on MEC service architecture.

**Figure 4:** MEC system application scenario.

**Figure 5:** Relationship between quality assurance, quality control, and quality assessment.

**Figure 6:** Area distribution diagram under the normal curve.

**Figure 7:** Hypothesis testing two types of error schematic diagram and quality control chart of two types of error loss.

**Figure 8:** Distribution of patients in the experiment in terms of gender and age.

**Figure 9:** Patient condition detection rate and detection accuracy.

**Figure 10:** Patients' satisfaction with the test and healthcare professionals' satisfaction with the test.

**Table 1:** Relationship between the test decision and the two types of errors (*L*_*o*_ is the null hypothesis).

	Conclusions based on sample observations	
Actual situation of overall distribution	Accept *L*_*o*_	Reject *L*_*o*_
*L*_*o*_ established	Correct judgment	1
*L*_*o*_ not established	2	Correct judgment

**Table 2:** Commonly used cumulative and (CUSUM) quality control rules.

Related parameters	Threshold values for starting accumulation and calculation	
Quality control rules	(T)	Quality control limits (h)
*C*_2.7*s*_^1.0*s*^	$\bar{x}\pm 1.0s$	±2.7*s*
*C*_3.0*s*_^1.0*s*^	$\bar{x}\pm 1.0s$	±3.0*s*
*C*_5.1*s*_^0.5*s*^	$\bar{x}\pm 0.5s$	±5.1*s*

**Table 3:** List of factors affecting the quality of clinical trials.

Quality control factor	Access to informed consent	Researcher compliance	Data logging	Outlier review	Subjects' compliance
Number of entries	2	9	4	5	2
Highest score	70	75	74	65	66
Lowest score	55	20	22	38	12

**Table 4:** Number of patients in each department in the second half of 2020.

	Men (number)	Women (number)
Surgery	499	33
Gynecology	—	256
Internal medicine	412	152
Other departments	390	148

## Data Availability

No data were used to support this study.
